The article "Serum Retinol Concentrations, Race, and Socioeconomic Status in of Women of Childbearing Age in the United States" was published in 2016. Journal: Nutrients.

# Serum Retinol Concentrations, Race, and Socioeconomic Status in of Women of Childbearing Age in the United States

**DOI:** 10.3390/nu8080508

**Published:** 2016-08-19

**Authors:** Corrine Hanson, Elizabeth Lyden, Chad Abresch, Ann Anderson-Berry

**Affiliations:** 1 College of Allied Health Professions, Medical Nutrition Education, University of Nebraska Medical Center, 984045 Nebraska Medical Center, Omaha, NE 68198-4045, USA; 2 College of Public Health, University of Nebraska Medical Center, 984375 Nebraska Medical Center, Omaha, NE 68198-4375, USA; elyden@unmc.edu; 3 CityMatCH, Annex 14, 4460 Farnam, Omaha, NE 68198-2170, USA; cabresch@unmc.edu; 4 Pediatrics, University of Nebraska Medical Center, 981205 Nebraska Medical Center, Omaha, NE 68198-1205, USA; alanders@unmc.edu

**Keywords:** vitamin A, women, childbearing, diet

## Abstract

Background: Vitamin A is an essential nutrient during pregnancy and throughout the lifecycle due to its role in the development of critical organ systems. Because maternal tissue is progressively depleted of vitamin A to supply fetal demands, women who become pregnant while possessing marginal vitamin A reserves are at increased risk of vitamin A inadequacy as pregnancy progresses. Few studies have assessed the relationship between socioeconomic factors and retinol status in women of childbearing age. Methods: We used the National Health and Nutrition Examination Survey (NHANES) to assess the relationship between serum retinol concentrations and socioeconomic factors in women of childbearing age. Women 14–45 years of age (*n* = 3170) from NHANES cycles 2003–2004 and 2005–2006 were included. Serum retinol concentrations were divided into categories according to World Health Organization criteria. All statistical procedures accounted for the weighted data and complex design of the NHANES sample. A *p*-value of < 0.05 was considered statistically significant. Results: The poverty score and race were significantly associated with vitamin A status after adjustment for confounders. Odds of retinol concentrations of <1.05 µmol/L were 1.85 times higher for those of lower socioeconomic status when compared to those of higher status (95% CI: 1.12–3.03, *p* = 0.02), and 3.1 times higher for non-Hispanic blacks when compared to non-Hispanic whites (95% CI: 1.50–6.41, *p* = 0.002). Dietary intakes of retinol activity equivalents were significantly lower in groups with higher poverty scores (*p* = 0.004). Conclusion There appear to be disparities in serum vitamin A levels in women of childbearing age related to income and race in the United States.

## 1. Introduction

Vitamin A is an essential nutrient throughout the lifecycle; however, its influence is particularly critical during periods when cells proliferate rapidly and differentiate, such as during pregnancy_._ Adequate vitamin A status in the mother is critical for fetal growth, morphogenesis, and maturation of multiple organ systems, including the immune system, lungs, and eyes [1,2]. Maternal vitamin A deficiency increases the risk of complications during pregnancy and in the postpartum period and has been positively associated with preterm delivery [3], maternal infections, night blindness, anemia [4], and birth defects [5]. Maternal vitamin A deficiency also has serious repercussions for the newborn and is associated with depressed immune function and higher morbidity and mortality due to infections [1], low birth weight [6], diaphragmatic hernia [7], bronchopulmonary dysplasia and other respiratory disease [8,9,10]. 

The article "Serum Retinol Concentrations, Race, and Socioeconomic Status in of Women of Childbearing Age in the United States" was published in 2016. Journal: Nutrients.

Vitamin A deficiency is one of the most prevalent and important nutritional deficiencies and has been known to be of public health significance in developing countries for several decades [11]. Worldwide, it affects 19 million pregnant women and is the underlying cause of 650,000 early childhood deaths annually [10]. The United States has been assumed to be free of vitamin A deficiency based on a high gross domestic product [12] and vitamin A status has only rarely been investigated in the US population, especially in women of childbearing age. Since there is no de novo fetal synthesis of vitamin A, the fetus relies completely on circulating maternal vitamin A. Signs of vitamin A deficiency may not be observed in the mother, but the rapidly developing fetus is more vulnerable to these effects [13]. Since maternal stores will be rapidly depleted in order to provide vitamin A to the developing fetus [14], it is critical that women of childbearing age are sufficient in vitamin A prior to conception. 

The National Health and Nutrition Examination Survey (NHANES) contains serum retinol concentrations and measures of socioeconomic status, allowing us to evaluate these relationships. Therefore, the objective of this study was to use NHANES data to examine the retinol status of women of childbearing age in the United States, and to assess the impact of poverty and race, as well as other indicators that have not previously been examined in this population, including food security and use of Supplemental Nutrition Assistance Programs (SNAP), on vitamin A status. 

## 2. Methods

Subjects: Women who were 14–45 years of age from NHANES the cycles 2003–2004 and 2005–2006 who were not missing serum retinol concentrations were included in the analysis. Serum retinol concentrations are not available in NHANES after 2006, and earlier waves were not included due to large amounts of missing data (up to 85%) on socioeconomic indices. The final number of eligible participants was 3710.

The article "Serum Retinol Concentrations, Race, and Socioeconomic Status in of Women of Childbearing Age in the United States" was published in 2016. Journal: Nutrients.

Outcomes: The main outcome variable was vitamin A status as assessed by serum retinol concentrations. Blood samples in NHANES were obtained by venipuncture and serum retinol was measured with the use of an isocratic, reversed-phase HPLC [15]. We categorized serum retinol concentrations into the following categories: ≤0.7, >0.7–1.05, and >1.05 based on guidelines from the World Health Organization [12] and other sources [16]. For the multivariate models, we dichotomized vitamin A status into insufficient (<1.05) and sufficient (>1.05). We chose these categories based on evidence that maternal stores will be rapidly depleted by the developing fetus [14], therefore we deemed it important that a woman begins a pregnancy with sufficient vitamin A stores. 

Dietary assessment: Dietary intake in the NHANES survey was determined from two interviewer-administered 24 h recalls using methodology developed and validated by the U.S. Department of Agriculture. The dietary recalls are conducted in English or Spanish in study participants who are 12 years and older. Three to 10 days later, all participants are asked to complete a second 24 h dietary recall interview by telephone. For this analysis, total nutrient intakes from the first day of 24 h recalls were used in order to limit the amount of missing data, which increased when both days were included. Study participants’ dietary intake of vitamin A in Retinol Activity Equivalents (RAE, mcg) per day was the main measure of vitamin A intake [17]. Intake of carotenoids in mcg, including alpha-carotene beta-carotene beta-cryptoxanthin, lycopene intake lutein + zeaxanthin were also assessed. Carotenes and beta-crytoxanthin have pre-vitamin A activity, and lutein + zeaxanthin and lycopene have been shown in the literature to potentially be important to the developing fetus [18,19]. 

Other covariates: Poverty to income ratio (PIR) was used as an index of socioeconomic status. We categorized PIR into ≤1.85 and >1.85 based on previous studies [20], or income that is 185% of the poverty threshold applied by the Food and Nutrition Service. The PIR is the ratio of household income to the poverty threshold after accounting for inflation and family size [21,22]. The PIR is used to determine eligibility for means-tested government-sponsored assistance programs relevant for women, particularly the Special Supplemental Nutrition Program for Women, Infants, and Children (WIC) [20]. Race/ethnicity was categorized as Hispanic, non-Hispanic white, non-Hispanic Black, and Other (including multi-racial). 

The article "Serum Retinol Concentrations, Race, and Socioeconomic Status in of Women of Childbearing Age in the United States" was published in 2016. Journal: Nutrients.

As inflammation is an important consideration in the evaluation of serum retinol concentrations [13], we adjusted for inflammation using serum concentrations of C-reactive protein (CRP). Estrogen use has also been found to be an important consideration in the evaluation of retinol concentrations in women [23] and was included in all models. To assess smoking status, survey participants were asked about current and past tobacco use. Smoking status was defined as: never, former (smoked >100 cigarettes in lifetime but does not currently smoke), and current (smoked >100 cigarettes in lifetime and smokes currently). Subject height and weight were measured during the clinical examination and were used to calculate body mass index (BMI). Other covariates included age and serum cholesterol [23].

Food insecurity was measured with the 18-item US Food Security Survey Module [24]. Questions are ordered by severity and attribute-related experiences or behaviors to insufficient resources to buy food over the past 12 months. A raw score was created by summing the affirmative responses of the 18 questions, with a higher score reflecting higher concentrations of food insecurity. Categories are then assigned on the basis of guidelines from the USDA: 0, full food security; 1–2, marginal food security; 3–5 (households without children) or 3–7 (households with children), low food security; and 6–10 (households without children) or 8–18 (households with children), very low food security. Food insecurity refers to households reporting low or very low food security. SNAP participation was assessed with the question, “in the last 12 months, did you or any members of your household receive Food Stamp benefits?” Both food insecurity and SNAP participation are measured at the household level [25].

Statistical Analysis: Descriptive statistics (counts and percentages and means and standard deviations) are shown for all participants. SAS version 9.4 (SAS, Cary, NC, USA) was used for all statistical analyses. Survey procedures in this software package incorporate sample weights and adjust analyses for the complex sample design of the survey. Survey sample weights were used in all analyses to determine estimates that were representative of the U.S. civilian, non-institutionalized population. The SAS procedures PROC SURVEYFREQ, PROC SURVEYMEANS, PROC SURVEYLOGISTIC and PROC SURVEYREG were used in computing descriptive analysis and doing regression analysis. The results of the descriptive analysis for categorical variables are represented by counts, percentages and weighted frequencies. Means, standard errors and 95% confidence intervals were used for continuous variables. Associations between categorical variables were determined using the Wald chi-square test which accounts for the complex survey design. *p*-values for the comparisons of continuous data between groups (e.g., retinol categories and PIR groups) were obtained from “PROC SURVEYREG” a SAS procedure that performs regression analysis for sample survey data. For the multivariate model, a backward selection method was used to determine the best subset of variables associated with vitamin A insufficiency. This method involved running a full model with all the predictors first and then sequentially removing factors that were least associated with the outcome until only variables significant at the *p* < 0.05 level were left in the final model. The full model included age, race/ethnicity, smoking status, BMI, CRP, total cholesterol, estrogen use, ratio of family income to poverty (dichotomized <1.85, ≥1.85), food stamps in the past 12 months, and food security category. A *p-*value of < 0.05 was considered statistically significant.

The article "Serum Retinol Concentrations, Race, and Socioeconomic Status in of Women of Childbearing Age in the United States" was published in 2016. Journal: Nutrients.

## 3. Results

The final number of eligible participants was 3710. Overall, the mean serum retinol concentration of the population was 1.79 µmol/L (SE: 0.01, 95% CI for mean: 1.76–1.81). The mean age of the participants was 30.1 years with a mean BMI of 26.6. Participants with a lower serum retinol had higher CRP and lower serum cholesterol concentrations than those with higher serum retinol concentrations. Lower serum retinol concentrations were also associated with poverty and race (Table 1). The overall prevalence of vitamin A deficiency in our cohort, as defined by serum retinol concentrations of ˂0.70 µmol/L, was very low at less than 1%. The overall prevalence of vitamin A insufficiency (>0.7–1.05) was 3.5%. The majority of the population (96.1%) was vitamin A sufficient with serum retinol concentrations >1.05 µmol/L. The demographic characteristics of the sample by serum retinol distribution are given in Table 1. 

The proportion of individuals who were vitamin A deficient or insufficient increased as poverty status increased (Table 2). Vitamin A intake was also significantly different between the socioeconomic groups, with those of lower socioeconomic status taking in an average of 93.9 less Retinal Activity Equivalents (RAE) when compared to the higher socioeconomic status group (464.7 mcg vs. 558.7 mcg, *p* = 0.004). Of the other carotenoids, only the intakes of lutein + zeaxanthin were significantly different between the two groups (*p* = 0.007) (Table 3). 

In the univariate analysis, a statistically significant association was seen between serum retinol concentrations and PIR (*p* < 0.001), race (*p* < 0.001), food security (*p* < 0.001), and use of Supplemental Nutrition Assistance Programs (SNAP) (*p* = 0.05). After adjusting for age, BMI, smoking status, serum cholesterol, CRP, and estrogen use, PIR and race maintained significant associations. For PIR, the odds of serum retinol concentrations of <1.05 were 1.85 times higher for those of lower socioeconomic status when compared to those of higher socioeconomic status (95% CI: 1.12–3.03, *p* = 0.02). The odds of serum retinol concentrations of <1.05 were 3.01 times higher for non-Hispanic blacks when compared to non-Hispanic whites (95% CI: 1.50–6.41, *p* = 0.002), and 2.68 times higher for “other race, including multi-race” vs. non-Hispanic whites (95% CI: 1.02–7.03, *p* = 0.04). The results of the multivariate analysis for all significant variables are shown in Table 4. 

The article "Serum Retinol Concentrations, Race, and Socioeconomic Status in of Women of Childbearing Age in the United States" was published in 2016. Journal: Nutrients.

## 4. Discussion

This study is among the first to examine a wide range of socioeconomic indicators, including SNAP use and food security, on retinol status in a nationally representative sample of women of childbearing age. Our study shows that lower poverty status and race increase the risk of suboptimal vitamin A stores in women of childbearing age in the United States. Because maternal tissues are progressively depleted of vitamin A to supply fetal demands [14], women who initially possess marginal or even adequate vitamin A stores at the beginning of pregnancy are at an increased risk of vitamin A inadequacy as pregnancy progresses. Radhika et al. found a significantly increased risk of spontaneous preterm delivery, maternal anemia, and pregnancy-induced hypertension when retinol levels were below 0.70 µmol/L, and based on those functional effects recommend a level of 0.70 µmol/L to define vitamin A deficiency in pregnancy [3]. Measurements of vitamin A concentrations in breast milk, maternal serum vitamin A concentration, and maternal dietary intake suggest that a maternal concentration of ≥1.05 µmol/L is necessary in order to maintain a sufficient vitamin A content in breast milk [26]. Therefore, it is imperative that women be vitamin A sufficient prior to becoming pregnant in order to avoid depletion of vitamin A stores due to fetal and lactation demands and subsequent ramifications to the mother or developing infant. 

Analysis of NHANES III (1988–1994) found that clinically low serum retinol concentrations were uncommon in USA adult residents [16]. However, racial differences did exist, with non-Hispanic black and Mexican American females being more likely than non-Hispanic white females to have low serum retinol concentrations [23]. Other limited survey information suggests that populations from poorer environments and with evidence of lower-quality dietary intakes in the United States do have a higher prevalence of lower serum retinol values [27,28]. Our analysis used the most recent NHANES cycles containing serum retinol information, and our findings also support an overall low prevalence of vitamin A deficiency and insufficiency during this time period. Our results also support the finding that there is not an even distribution of vitamin A status across ethnic, racial, and socioeconomic strata. It would appear that this finding does have implications for the woman in her childbearing years, through pregnancy, and eventually impacting the newborn infant, as studies have shown that infants born in lower socioeconomic groups have lower cord retinol values as compared to neonates of higher-income and better-educated families [28,29].

The article "Serum Retinol Concentrations, Race, and Socioeconomic Status in of Women of Childbearing Age in the United States" was published in 2016. Journal: Nutrients.

The primary cause of vitamin A deficiency is inadequate dietary intake, especially with diets that are of poor quality or diversity. Vitamin A is a fat-soluble vitamin that can be obtained from the diet in two forms, preformed vitamin A or pro-vitamin A compounds. Preformed vitamin A includes retinol which can be found in animal sources such as dairy products, fish, meat, and eggs and comprises up to 70% of the daily vitamin A intake in the United States [30]. Pro-vitamin A compounds are precursors for retinol and include β-carotene, α-carotene, and β-cryptoxanthin [2]. These must be obtained from the diet and are found primarily in fruits and vegetables [2]. Pro-vitamin A compounds provide more than 30% of the daily vitamin A intake in the United States [2]. Recent studies have raised concerns regarding nutrient intake in the United States, especially with regard to vitamin A and vitamin A precursors from fruits and vegetables. Data from 2003 to 2008 NHANES cycles demonstrate that women of childbearing age in the United States are not meeting nutrient guidelines for vitamin A intake, with distinct differences present between ethnic groups and socioeconomic strata [20,31,32]. Lower income individuals consumed lower quality foods when compared to those with higher incomes, including fruits and vegetables, as measured by the Alternate Healthy Eating Index [33]. 

Multiple factors contribute to low-income individuals having a high risk of poor quality diet, including lack of access to grocery stores and the high cost of healthy foods [34]. Individuals in the lowest income households are the least likely to consume vegetables and fruits [25,35,36], which are the primary sources of pro-vitamin A compounds, and are more likely to consume foods high in fat and sugar and low in fiber [37,38]. In addition to socioeconomic status, racial and ethnic minority groups experience diet-related disparities, and consequently tend to have poorer nutrient profiles and dietary patterns relative to whites. These disparities also include diets low in fruits and vegetables. According to the Behavioral Risk Factor Surveillance Survey, only 19% of Hispanics and 22% of African Americans consume vegetables ≥3 times per day, the lowest of any USA racial or ethnic groups [35]. Results from NHANES III (1999–2002) show that non-Hispanic blacks were 43% and Hispanics were 5% less likely than whites to meet USDA fruit and vegetable guidelines [39]. This data raises significant concerns that access to nutritional foods is not evenly distributed, and as a result, there are likely populations at risk for nutritional deficiencies.

The article "Serum Retinol Concentrations, Race, and Socioeconomic Status in of Women of Childbearing Age in the United States" was published in 2016. Journal: Nutrients.

Use of prenatal vitamins may not be a contributing factor toward closing the gap in retinol status by socioeconomic group, as pre-conception use of multivitamins in the United States is often poor. Only 23% of women of childbearing age take a prenatal vitamin, which is an important source of nutrients critical during the pre-conception period, including vitamin A [40]. This number has not increased despite the Healthy People 2020 goal that 80% of women of childbearing age will consistently use a prenatal vitamin supplement [41]. Data from the Midwestern region of the United States shows only 25.2% of black women take a prenatal vitamin, as opposed to 46.7% of white women [41]. This gap is even more distinct by poverty status, as only 26% of women below 200% of the Federal Poverty Limit (FPL) take a prenatal vitamin, as opposed to 61% who are above 200% FPL [40]. 

We also investigated the impact of other socioeconomic indicators on vitamin A status that have not been well explored, including food insecurity and SNAP use. Food insecurity, or lack of access to “enough food for an active, healthy life”, as defined by the USDA, is common among the urban poor and may have important health implications. Other studies have shown that adults reporting insecurity about the availability of nutritious food had 32% increased odds of being obese compared to adults reporting security in access to nutritious food [42]. While we did find an association between food security and retinol status in the univariate analysis, this was significantly attenuated after adjustment for confounders, suggesting that other factors, such as income, may be of more relevance. We also evaluated serum retinol concentrations in relation to SNAP use, as other studies have also shown that SNAP participants may have lower diet quality and intakes of fruits and vegetables when compared to income-eligible nonparticipants [25]; however, our study did not translate these findings into an impact on serum retinol levels. 

The article "Serum Retinol Concentrations, Race, and Socioeconomic Status in of Women of Childbearing Age in the United States" was published in 2016. Journal: Nutrients.

Our study has several limitations. The cross-sectional nature of NHANES makes it difficult to infer any causation, and it is also possible that confounding occurred from variables not considered in our analysis. Additionally, dietary intake in NHANES is based on 24 h recalls, which may be unlikely to be representative of usual intake, as day-to-day intake of fruits and vegetables can be highly variable. However, a single 24 h recall is adequate for estimates of group means [43]. Additionally, we did not assess the zinc status of the population. Reductions in retinol binding protein have been reported with moderate zinc restriction [2]; therefore, zinc status may impact the amount of retinol that can circulate. Plasma zinc levels were not available for these NHANES cycles, limiting our ability to assess the zinc status of the population. Serum retinol levels are also under tight homeostatic control and may not be reliable indicators of the vitamin A status of an individual [44]. Our use of the WHO retinol classifications, however, does provide us with information about the vitamin A status of this important population [44], women of childbearing age. 

## 5. Conclusions

Our results demonstrate it is possible that vitamin A deficiency is a public health concern in nutritionally disadvantaged populations of industrialized societies. More research is needed to determine what type of interventions will be best for specific populations, especially the low-income and minority populations that bear a greater burden of vitamin A inadequacy. As the population of the United States becomes more diverse [45], issues regarding health and disparities in the diet become even more salient. 

## Figures and Tables

**Table 1:** Participant characteristics by serum retinol category.

	Serum Retinol Category, µmol/L Mean (SE)			
Characteristic	≤0.7 (*n* = 18)	>0.7–1.05 (*n* = 240)	>1.05 (*n* = 3452)	*p*-Value
Continuous variables Mean (SD)				
Age, year	29.5 (4.3)	27.2 (.090)	30.2 (0.2)	<0.0001
BMI	27.0 (2.0)	29.6 (0.76)	27.1 (0.2)	<0.0001
Socioeconomic Status (poverty:income ratio)	2.1 (0.6)	1.9 (0.1)	2.8 (0.06)	<0.0001
C-Reactive protein (mg/dL)	1.2 (0.6)	0.9 (0.2)	0.4 (0.01)	0.009
Energy intake (kcals/day)	2054.1 (213.1)	1914.6 (89.1)	1975.6 (15.8)	0.78
Vitamin A intake (RAE, mcg)	440.7 (112.5)	414.3 (57.5)	529.5 (12.1)	0.14
Αlpha-carotene intake (mcg)	367.2 (262.3)	227.8 (53.5)	325.7 (30.1)	0.23
Beta-carotene intake (mcg)	1568.9 (922.3)	1547.0 (615.9)	1613.1 (73.6)	0.99
Beta-cryptoxanthin intake (mcg)	92.1 (52.1)	152.2 (24.9)	115.0 (6.3)	0.26
Lycopene intake (mcg)	2530.8 (1134.1)	5302.7 (769.6)	5063.3 (201.2)	0.11
Lutein + zeaxanthin intake (mcg)	1221.6 (412.0)	1202.4 (407.6)	1092.2 (50.5)	0.92
Serum cholesterol (mg/dL)	165.3 (21.4)	174.4 (3.6)	188.2 (1.0)	0.002
Discrete variables	N (%)			
Race				<0.0001
Hispanic	5 (0.14)	73 (5.2)	1068 (94.7)	
Non-Hispanic White	5 (0.34)	47 (1.8)	1364 (98.0)	
Non-Hispanic Black	7 (1.3)	108 (9.7)	858 (89.9)	
Other	1 (1.3)	12 (4.5)	162 (94.2)	
Smoking				*
Never	13 (0.7)	93 (3.7)	1327 (95.6)	
Former	0	19 (2.7)	309 (97.3)	
Current	0	19 (2.5)	462 (97.5)	
Unknown	5 (0.2)	109 (4.7)	1354 (95)	
Supplemental Nutrition				<0.0001
Assistance Program				
Yes	5 (0.5)	50 (8.3)	434 (91.2)	
No	13 (0.4)	186 (2.9)	2972 (96.7)	
Food Security				0.05
Full	8 (0.3)	150 (2.9)	2371 (96.7)	
Marginal	4 (0.4)	37 (6.6)	412 (93)	
Low	4 (0.2)	27 (4.4)	383 (94.6)	
Very Low	2 (0.2)	21 (5.1)	213 (94.7)	
Supplemental Estrogen				*
Use				
Yes	0	5 (0.7)	449 (99.3)	
No	12 (0.5)	125 (3.9)	1723 (95.6)	

* *p*-value non-calculable due to zeros.

The article "Serum Retinol Concentrations, Race, and Socioeconomic Status in of Women of Childbearing Age in the United States" was published in 2016. Journal: Nutrients.

**Table 2:** Proportion of participants in each vitamin A category, by PIR.

Poverty Group (PIR)	Serum Retinol Category, µmol/L	N (%)	*p*-Value
≤1.85	≤0.7	12 (0.4)	<0.0001
	0.7 ≤ 1.05	137 (5.9)	
	>1.05	1646 (93.5)	
>1.85	<0.7	5 (0.3)	
	0.7 ≤ 1.05	94 (2.0)	
	>1.05	1654 (97.7)	

**Table 3:** Intake of vitamin A and carotenoids by PIR group.

Nutrient	Intakes in PIR ≤ 1.85 Group Mean (SE) *n* = 1710	Intakes in PIR ˃ 1.85 Group Mean (SE) *n* = 1701	*p*-Value
Vitamin A, RAE (mcg)	464.7 (21.0)	558.7 (13.1)	0.004
Alpha-carotene (mcg)	349.8 (75.0)	312.3 (26.1)	0.64
Beta-carotene (mcg)	1530.4 (178.9)	1671.4 (67.6)	0.47
Beta-cryptoxanthin (mcg)	123.7 (8.8)	112.1 (8.6)	0.33
Lycopene (mcg)	5488.1 (436.9)	4870.6 (200.3)	0.19
Lutein + zeaxanthin (mcg)	942.7 (75.0)	1200.8 (64.3)	0.007

**Table 4:** The risk of serum retinol of less than 1.05 µmol/L for variables significant in multivariate analysis.

Category	OR	95% CI	*p*-Value
Socioeconomic status (Poverty:income ratio of ≤1.85 vs. >1.85)	1.85	1.12–3.03	0.02
Race (Non-Hispanic Black vs. Non-Hispanic White)	3.01	1.50–6.41	0.002
Race (Other Race—Including Multi-Racial vs. Non-Hispanic White)	2.68	1.02–7.03	0.04
Smoking (Current vs. Never)	0.48	0.24–0.99	0.04
Cholesterol	0.99	0.98–1.00	0.04
Estrogen Use (Yes vs. No)	0.17	0.05–0.50	0.003
C-Reactive Protein	1.55	1.34–1.78	<0.001
